# Effect of Nursing Method of Psychological Intervention Combined with Health Education on Lung Cancer Patients Undergoing Chemotherapy

**DOI:** 10.1155/2022/2438612

**Published:** 2022-02-16

**Authors:** Jing Yu, Ting Huang, Jing Xu, Jing Xiao, Qing Chen, Lixia Zhang

**Affiliations:** Internal Medicine-Oncology,Wuhan Fourth Hospital, Puai Hospital, Tongji Medical College, Huazhong University of Science and Technology, Wuhan 430034, Hubei Province, China

## Abstract

At present, lung cancer has become clinically the malignant tumor with the highest incidence and mortality rate in China. Smoking, environmental pollution, infection, etc., are closely related to lung cancer. To investigate the effect of the nursing method of psychological intervention combined with health education on lung cancer patients undergoing chemotherapy, 70 lung cancer patients who received chemotherapy in our hospital from June 2017 to June 2020 were selected and randomly divided into a routine intervention group (*n* = 35) and a combined intervention group (*n* = 35). Patients in the two groups had the same chemotherapy method and medication. The routine intervention group received the routine nursing intervention, while on this basis, the combined intervention group received psychological intervention combined with health education. After 6-week nursing, self-rating anxiety scale (SAS) score, self-rating depression scale (SDS) score, cancer pain score before and after nursing, improvement of respiratory function before and after nursing, sleep quality score, quality of life score, and nursing satisfaction were analyzed. Through nursing intervention, the quality of life indexes such as physiological, physical, social, emotional, and other indexes in the combined intervention group were significantly better than those in the routine intervention group, with statistical differences (*P* < 0.01). The nursing satisfaction in the combined intervention group was significantly better than that in the routine intervention group, with statistical significance (*χ*^2^ = 8.9342, *P* < 0.05). The psychological intervention combined with health education for lung cancer patients undergoing chemotherapy can effectively alleviate anxiety and depression, increase confidence in treatment, reduce pain and significantly improve sleep quality, respiratory function, quality of life, and nursing satisfaction.

## 1. Introduction

In recent years, with the development of society and the change of lifestyle, the incidence of lung cancer has been increasing year by year. At present, lung cancer has become clinically the malignant tumor with the highest incidence and mortality rate in China [1]. Smoking, environmental pollution, infection, etc., are closely related to lung cancer. The clinical manifestations of lung cancer patients mainly include cough, expectoration, hemoptysis, and chest pain and tightness, seriously affecting patients' quality of life [2, 3]. In clinical treatment, patients with advanced lung cancer can mainly receive surgical treatment and conservative chemotherapy. However, with killing cancer cells, chemotherapy also kills a large number of healthy cells, resulting in serious side effects such as weakened immunity, organ function impairment, nausea, vomiting, fatigue, alopecia, etc. [4, 5]. Due to the physiological pain caused by chemotherapy and the disease itself, as well as the critical condition and long course of the disease, patients have poor sleep quality and negative emotions such as anxiety, fear, depression, etc., which further aggravates the patients' condition and reduces the treatment effect [6]. Some studies have found that psychological intervention for lung cancer patients can effectively alleviate their negative emotions and improve their treatment compliance [7]. Health education for lung cancer patients can raise the awareness of lung cancer-related knowledge, effectively reduce cancer pain, and improve the quality of life [8]. The main ways to treat lung cancer patients clinically include surgical treatment, chemotherapy, radiotherapy, etc. Chemotherapy is an effective method by killing cancer cells with chemical drugs to treat cancer, reduce and inhibit the metastatic lesions of cancer [9]. In this study, 70 lung cancer patients who received chemotherapy in our hospital from June 2017 to June 2020 were selected, and the nursing effect of psychological intervention combined with health education on lung cancer patients undergoing chemotherapy was analyzed. The results are as follows.

## 2. Materials and Methods

### 2.1. General Information

70 lung cancer patients who received chemotherapy in our hospital from June 2017 to June 2020 were selected and randomly divided into a routine intervention group (*n* = 35) and a combined intervention group (*n* = 35). This study was approved by the Hospital Ethics Committee, and all patients were informed of the process of this study, voluntarily participated in, and signed the informed consent. In this study, the proportion of male and female was 19 : 16 in the routine intervention group wherewith the average age of (48.45 ± 4.28) years old, patients aged from 23 to 78 years old, including 15 patients with adenocarcinoma, 12 patients with squamous cell carcinoma, and 8 patients with small cell carcinoma. The proportion of male and female was 20 : 15 in the combined intervention group, with an average age of (48.72 ± 4.37) years old, patients aged from 22 to 81 years old, including 14 patients with adenocarcinoma, 14 patients with squamous cell carcinoma, and 7 patients with small cell carcinoma. There were no statistical differences in general information such as gender, age, etc., in the two groups, with comparability (*P* > 0.05).

### 2.2. Inclusion/Exclusion Criteria

#### 2.2.1. Inclusion Criteria

1. Patients were diagnosed with lung cancer by pathological examination.
2. Patients had high treatment compliance.
3. Patients had stable vital signs.
4. Patients had no disturbance of consciousness, communication barriers, and psychiatric history.
5. Patients had Karnofsky performance status (KPS) score (≥60 points).

#### 2.2.2. Exclusion Criteria

1. Patients had incomplete clinical data.
2. Patients needed for surgical treatment.
3. Patients had a KPS score (<60 points).
4. Patients had insufficient treatment cooperation.
5. Patients had severe organic diseases in the heart, liver, kidney, etc.

### 2.3. Methods

The lung cancer patients in the two groups were given the same chemotherapeutic drugs (3 weeks as a course of treatment, a total of 2 courses of intervention).

Patients in the routine intervention group received the routine nursing intervention, mainly including routine pathography, vital signs monitoring, medication, and dietary guidance. Additionally, infection prevention and targeted care for side effects such as alopecia and phlebitis caused by chemotherapy were also carried out.

Patients in the combined intervention group received psychological intervention combined with health education on the basis of the treatment in the routine intervention group. The specific details are as follows.

1. Psychological intervention. With the long course of the disease, severe cancer pain, and side effects of chemotherapy, lung cancer will lead to negative emotions such as fear, anxiety, and depression in lung cancer patients undergoing chemotherapy, greatly reducing the treatment effect. Nursing staff should communicate with patients closely, grasp their psychological state in real-time, and adjust their bad moods in time. In addition, according to the patients' own educational level and condition, targeted interventions such as more relative accompany, entertainment programs, etc., should be given to alleviate patients' negative emotions, and publicizing successful cases in daily communication should also be given to enhance patients' confidence in healing.
2. Health education. Nursing staff should educate patients and their families about lung cancer according to their own conditions, with common and easy-to-understand language, so as to clarify the pathogenesis of cancer, measures of alleviating cancer pain, treatment methods, and mechanisms of lung cancer, diet, medication, exercise, etc. Additionally, nursing staff should also clarify the positive role of good psychological and physical status in improving the therapeutic effect and improving the treatment cooperation of patients. The propaganda and education of the health education should be carried out 3 to 4 times a week. Specific measures include the issuance of health hand cards, lectures on health, one-to-one answers, and other forms. During the propaganda, the family members of patients are also encouraged to participate together to raise the awareness of lung cancer disease and nursing skills.

### 2.4. Observation Indexes

SAS score was adopted to evaluate the anxiety degree of lung cancer patients, and a lower score indicated a better result. SDS score was used to evaluate the depression degree of lung cancer patients, and a lower score indicated a better result. Numeric rating scales (NRS) were used to evaluate the cancer pain of lung cancer patients before and after nursing, and a lower score indicated a better result. Respiratory function indexes including respiratory rate (RP), oxygen saturation (SaO_2_), maximal voluntary ventilation (MVV), minute ventilation volume (MV), and forced expiratory volume in one second (FEV1) in the two groups were all detected before and after nursing. Pittsburgh sleep quality index (PSQI) was adopted to evaluate the sleep quality of lung cancer patients before and after nursing, and a lower score indicated a better result. SF-36 scale was used to evaluate the quality of life of lung cancer patients, mainly including physiological, physical, social, emotional, and other indexes and a higher score indicated a better result. Nursing satisfaction was evaluated by a self-made nursing satisfaction questionnaire in our hospital, which was filled out by patients after nursing, and the evaluation criteria were divided into very satisfied, rather satisfied, satisfied and unsatisfied.

### 2.5. Statistical Treatment

SPSS18.0 software was adopted to statistically process and analyze the relevant materials and data in this study. The measurement data were expressed as $\left(\bar{x}\pm s\right)$, and tested by *t*-test. The enumeration data were expressed as [*n* (%)] and tested by *X*^2^ test. The differences had statistical significance when *P* < 0.05.

## 3. Results

### 3.1. Comparison of SAS Score and SDS Score before and after Care of the Two Groups of Patients

Before nursing, there were no statistical differences in SAS score and SDS score in the two groups (*P* > 0.05). After nursing, the SAS score and SDS score in the combined intervention group were significantly better than those in the routine intervention group, with statistical differences (*P* < 0.05). Specific details can be seen in Figure 1.

Note: Figure 1 Comparison of SAS score and SDS score before and after care of the two groups of patients. The abscissa represents SAS score before nursing, SAS score after nursing, SDS score before nursing, and SDS score after nursing, while the ordinate represents the score. It can be seen from Figure 1 that there were no significant differences in SAS score and SDS score in the two groups before nursing. After nursing, the SAS score in the routine intervention group was higher than that in the combined intervention group, and the SDS score in the routine intervention group was higher than that in the combined intervention group, with significant differences.

### 3.2. Comparison of NRS Scores before and after Care of the Two Groups of Patients

Before nursing, there were no statistical differences in NRS scores in the two groups (*P* > 0.05). After nursing, the NRS score in the combined intervention group was significantly better than that in the routine intervention group, with statistical differences (*P* < 0.05). The specific details can be seen in Figure 2.

The abscissa represents the NRS score before and after nursing, while the ordinate represents the score. It can be seen from Figure 2 that there were no significant differences in NRS score in the two groups before nursing, and after nursing, the NRS score in the routine intervention group was higher than that in the combined intervention group, with significant differences.

### 3.3. Comparison of the Improvement of Respiratory Function in the Two Groups before and after Nursing

Before nursing, there were no significant differences in the respiratory function indexes such as RR, SaO2, MVV, MV, FEV1, etc., in the two groups (*P* > 0.05). After nursing, there was no significant difference in SaO2 in the two groups (*P* > 0.05), and RR, MVV, MV, FEV1, etc., in the combined intervention group were significantly better than those in the routine intervention group, with statistical differences (*P* < 0.05). The specific details can be seen in Table 1.

### 3.4. Comparison of Patients' Sleep Quality Index (PSQI) Scores before and after Care in the Two Groups

Before nursing, there were no statistical differences in PSQI scores in the two groups (*P* > 0.05). After nursing, the PSQI score in the combined intervention group was significantly better than that in the routine intervention group, with statistical differences (*P* < 0.05). The specific details can be seen in Figure 3.

The abscissa represents PSQI score before nursing and PSQI score after nursing, while the ordinate represents the score. As shown in Figure 3, there were no significant differences in PSQI scores in the two groups before nursing. After nursing, the PSQI score in the routine intervention group was higher than that in the combined intervention group, with significant differences.

### 3.5. Comparison of Patients' Quality of Life Scores in the Two Groups

Through nursing intervention, the quality of life indexes such as physiological, physical, social, emotional, and other indexes in the combined intervention group were significantly better than those in the routine intervention group, with statistical differences (*P* < 0.01). The specific details can be seen in Table 2.

### 3.6. Comparison of Nursing Satisfaction in the Two Groups

Nursing satisfaction in the combined intervention group was significantly better than that in the routine intervention group, with statistical significance (*χ*^2^ = 8.9342, *P* < 0.05). The specific details can be seen in Table 3.

## 4. Discussion

With the characteristics of high morbidity and mortality, lung cancer is one of the common malignant tumors, and its pathogenesis is closely related to daily habits, social environment, and other factors, which causes severe physiological pain to patients, thus seriously threatening patients' life safety [10]. The main ways to treat lung cancer patients clinically include surgical treatment, chemotherapy, radiotherapy, etc. Chemotherapy is an effective method by killing cancer cells with chemical drugs to treat cancer, reduce and inhibit the metastatic lesions of cancer [9]. Smoking, environmental pollution, infection, etc., are closely related to lung cancer. The clinical manifestations of lung cancer patients mainly include cough, expectoration, hemoptysis, and chest pain and tightness, seriously affecting patients' quality of life [2, 3]. Chemotherapy is administered systemically, which will lead to a variety of toxic and side effects in lung cancer patients undergoing chemotherapy, such as alopecia, fatigue, weakness, sleep disorders, nausea and vomiting, impaired liver and kidney function, myelosuppression, etc. [11]. Some studies have found that psychological intervention for lung cancer patients can effectively alleviate their negative emotions and improve their treatment compliance [7]. Because of the pain of lung cancer and the toxic side effects of chemotherapy, lung cancer patients will have negative emotions such as anxiety, depression, etc., which will reduce the confidence in treatment and treatment compliance, thus ultimately affecting the treatment effect. Psychological intervention for lung cancer patients undergoing chemotherapy is one of the common interventions in clinical nursing, which can effectively address patients' concerns, correct misconceptions, greatly alleviate negative emotions, enhance treatment confidence, enthusiasm as well as compliance, thus further improving the clinical efficacy [12, 13]. In recent years, some studies have reported that health education intervention for lung cancer patients undergoing chemotherapy can effectively raise the awareness of the pathogenesis and occurrence of the disease and can clarify the treatment plan and prognostic methods, thus significantly eliminating the uncertainty of lung cancer treatment, enhancing treatment confidence, and having positive significance for clinical treatment [14, 15].

In this study, 70 lung cancer patients who received chemotherapy in our hospital from June 2017 to June 2020 were selected to investigate the nursing effect of psychological intervention combined with health education on lung cancer patients undergoing chemotherapy. The result showed that after the nursing intervention, the SAS score and SDS score in the combined intervention group were significantly better than those in the routine intervention group, demonstrating that psychological intervention combined with health education can effectively alleviate patients' anxiety. The NRS score and PSQI score in the combined intervention group were significantly better than those in the routine intervention group, revealing that the combined intervention can effectively reduce the degree of cancer pain and improve patients' sleep quality. Some studies have shown that psychological intervention combined with health education can improve patients' cognitive level of cancer, alleviate their anxiety and depression, as well as effectively improve their cancer pain and sleep quality, having a positive significance in improving the quality of life and treatment effect [16, 17]. In the evaluation of the respiratory function indexes in the two groups after the nursing intervention, it was found that the respiratory function indexes such as RR, MVV, MV, and FEV1, as well as the quality of life indexes such as in physiological, physical, social, emotional, and other indexes in the combined intervention group were significantly better than those in the routine intervention group, thus demonstrating that the combined intervention can effectively improve patients' respiratory function, alleviate their clinical symptoms such as dyspnea and tachypnea, as well as improve the quality of life. There were consistent results between the study and *Effect of a Web-based Health Education Program on Quality of Life and Symptom Distress of Initially Diagnosed Advanced Non-Small Cell Lung Cancer Patients: A Randomized Controlled Trial* written by Lin Y. E. et al.' s [18] and others. It was mentioned in this study that the propaganda and education of health education for lung cancer patients to improve their self-regulation skills can effectively improve lung function, relieve dyspnea, tachypnea, and other clinical symptoms, and reduce the degree of cancer pain, anxiety, and depression, significantly improving the quality of life. Studies have shown that the key to successful psychological intervention is to improve the nurse-patient relationship to enhance the trust and dependence of patients on nursing staff, which can positively raise patients' awareness of disease and treatment cooperation [19, 20]. In the study, nurses were required to communicate and interact with patients closely, grasp patient's own conditions and the changes of their psychological state in time, and show respect and enthusiasm for patients during the process of communication so as to enhance patients' enthusiasm for cooperating with nursing staff in treatment. This study found that the nursing satisfaction in the combined intervention group was significantly better than that in the routine intervention group, confirming that close communication with patients can effectively improve the nurse-patient relationship and patients' treatment compliance, thus achieving the goal of smoothly treating lung cancer.

## 5. Conclusion

In conclusion, the psychological intervention combined with health education has a positive nursing effect on lung cancer patients undergoing chemotherapy, which can effectively improve negative emotions such as anxiety and depression, alleviate cancer pain, and significantly improve sleep quality, respiratory function, clinical symptoms, quality of life, and nursing satisfaction, playing a positive role in improving nurse-patient relationship, enhancing confidence in the treatment and improving clinical efficacy; and it is worthy of clinical popularization and application. However, there are still limitations in this study, and the experimental subjects are not sufficient. More experiments are needed to verify the experimental conclusions in the future.

## Figures and Tables

**Figure 1:** Comparison of SAS score and SDS score before and after care of the two groups of patients.

**Figure 2:** Comparison of NRS scores before and after care of the two groups of patients.

**Figure 3:** Comparison of PSQI scores before and after care in the two groups.

**Table 1:** Comparison of the improvement of respiratory function in the two groups before and after nursing.

Indexes		Combined intervention group (*n* = 35)	Routine intervention group (*n* = 35)	*t*	*p*
RR (time/min)	Before nursing	19.74 ± 5.28	19.67 ± 5.36	0.055	>0.05
	After nursing	12.24 ± 3.89	17.58 ± 5.14	4.901	<0.01
SaO_2_ (%)	Before nursing	86.87 ± 20.82	87.05 ± 20.93	0.036	>0.05
	After nursing	96.15 ± 28.63	90.83 ± 29.41	0.767	>0.05
MVV (L)	Before nursing	48.86 ± 14.27	49.07 ± 13.96	0.062	>0.05
	After nursing	69.27 ± 20.26	51.36 ± 16.21	4.084	<0.01
MV (L/min)	Before nursing	1.85 ± 0.49	1.87 ± 0.52	0.166	>0.05
	After nursing	3.05 ± 0.68	2.15 ± 0.63	5.744	<0.01
FEV1 (L)	Before nursing	0.93 ± 0.23	0.92 ± 0.21	0.190	>0.05
	After nursing	1.57 ± 0.39	1.07 ± 0.27	6.236	<0.01

**Table 2:** Comparison of patients' quality of life scores in the two groups.

Group	Physiological index	Physical index	Social index	Emotional index
Routine intervention group (*n* = 35)	60.4 ± 2.2	60.3 ± 2.2	64.3 ± 2.6	61.3 ± 2.3
Combined intervention group (*n* = 35)	77.8 ± 2.5	79.7 ± 2.0	81.3 ± 3.0	78.5 ± 2.6
*t*	30.911	38.602	25.334	29.314
*p*	<0.01	<0.01	<0.01	<0.01

**Table 3:** Comparison of nursing satisfaction in the two groups.

Group	Very satisfied	Rather satisfied	Satisfied	Unsatisfied	Satisfaction
Routine intervention group (*n* = 35)	7	12	4	12	65.71%
Combined intervention group (*n* = 35)	10	17	6	2	94.29%
*χ* ^2^					8.9342
*p*					<0.05

## Data Availability

The datasets used and/or analyzed during the current study are available from the corresponding author on reasonable request.

## References

[1] Tanaka I., Morise M., Miyazawa A. (2020). Potential benefits of bevacizumab combined with platinum-based chemotherapy in advanced non-small-cell lung cancer patients with EGFR mutation. *Clinical Lung Cancer*.

[2] Rana R. H., Alam F., Alam K., Gow J. (2020). Gender-specific differences in care-seeking behaviour among lung cancer patients: a systematic review. *Journal of Cancer Research and Clinical Oncology*.

[3] Ishii H., Azuma K., Kawahara A., Matsuo N., Tokito T., Hoshino T. (2020). Atezolizumab plus carboplatin and etoposide in small cell lung cancer patients previously treated with platinum-based chemotherapy. *Investigational New Drugs*.

[4] Quist M., Langer S. W., Lillelund C. (2020). Effects of an exercise intervention for patients with advanced inoperable lung cancer undergoing chemotherapy: a randomized clinical trial. *Lung Cancer*.

[5] Thiesing L. C., Karg N., Brückl W., Würflein D., Ficker J. H., Parsch W. (2020). Predictors and effects of reduced chemotherapy dosing in patients with non-small cell lung cancer IIIB. *Pneumologie*.

[6] Christina Huang W., James W., Gino C. (2020). Association of cancer center type with treatment patterns and overall survival for patients with sacral and spinal chordomas: an analysis of the National Cancer Database from 2004 to 2015. *Journal of Neurosurgery. Spine*.

[7] Toshiko K., Shigetoshi Y., Mariko T. (2020). Immunological features of a lung cancer patient achieving an objective response with anti-programmed death-1 blockade therapy. *Cancer Science*.

[8] Corsini E. M., Annikka W., Apar P., Zhou N., Antonoff M. B., Hofstetter W. L., Mehran R. J. (2021). Pathological nodal disease defines survival outcomes in patients with lung cancer with tumour major pathological response following neoadjuvant chemotherapy. *European Journal of Cardio-Thoracic Surgery*.

[9] D’Almeida Preto D., Baston M. T., Geraige C. C. (2019). Impact of AferBio® on quality of life and chemotherapy toxicity in advanced lung cancer patients (AFERBIO study): protocol study for a phase II randomized controlled trial. *BMC Cancer*.

[10] Jianzhong W., Yanjun C., Respiratory D. O. (2019). Staged cognitive behavior management in the negative psychological state of lung cancer chemotherapy. *China Continuing Medical Education*.

[11] Dapkeviiūt A., Dakeviiūt A., Zablockis R. (2019). Association between the Khorana score and pulmonary embolism risk in patients with advanced stage lung cancer. *The Clinical Respiratory Journal*.

[12] Jazieh A., Alkaiyat M. O., Ali Y., Hashim M. A., Abdelhafiz N., Al Olayan A. (2019). Improving adherence to lung cancer guidelines: a quality improvement project that uses chart review, audit and feedback approach. *Nephron Clinical Practice*.

[13] Hesketh P. J., Palmas M., Nicolas P. (2018). Preventing chemotherapy-induced nausea and vomiting in patients with lung cancer: efficacy of NEPA (netupitant-palonosetron), the first combination antiemetic. *Supportive Care in Cancer Official Journal of the Multinational Association of Supportive Care in Cancer*.

[14] Pelizzari G., Cortiula F., Giavarra M. (2020). Platinum-Based Chemotherapy in Older Patients with Non-small Cell Lung Cancer: What to Expect in the Real World. *Drugs & Aging*.

[15] Moosavi S., Rohani C., Borhani F., Akbari M. E. (2020). Spiritual Care Experiences by Cancer Patients, Their Family Caregivers and HealthCare Team Members in Oncology Practice Settings: A Qualitative Study. *Explore*.

[16] Mitchell K. R., Brassil K. J., Fujimoto K., Fellman B. M., Shay L. A., Springer A. E. (2020). Exploratory factor Analysis of a patient-centered cancer care measure to support improved assessment of patients’ Experiences. *Value in Health*.

[17] Tian S., Saravanan K., Mothana R. A., Ramachandran G., Rajivgandhi G., Manoharan N. (2020). Anti-cancer Activity of Biosynthesized Silver Nanoparticles Using *Avicennia marina* against A549 Lung Cancer Cells through ROS/mitochondrial damages. *Saudi Journal of Biological ences*.

[18] Lin Y. E., Huang C. C., Kuo H. P., Chen S. C. (2019). Effects of a web-based health education program on quality of life and symptom distress of initially diagnosed advanced non-small cell lung cancer patients: a randomized controlled trial. *Journal of Cancer Education*.

[19] Liang Z., Rui W., Min N., Jing Z., Xulei G., Qiaoyun L. (2018). Effect of health education by feedback method on health literacy level of lung cancer patients undergoing operation. *Chinese Community Doctors*.

[20] Mingshu W., Jinzhi X. U., Oncology D. O. (2018). The effect of the human mind mapping for the compliance of whole course of health education in non-small cell lung cancer patients. *China Journal of Health Psychology*.

